# An Ultrasonic-Based Sensor System for Elderly Fall Monitoring in a Smart Room

**DOI:** 10.1155/2022/2212020

**Published:** 2022-11-07

**Authors:** Chokemongkol Nadee, Kosin Chamnongthai

**Affiliations:** Department of Electronic and Telecommunication Engineering, Faculty of Engineering, King Mongkut's University of Technology, Thonburi, Bangkok, Thailand

## Abstract

To reduce the risk of elderly people falling in a private room without relying on a closed-circuit television system that results in serious privacy and trust concerns, a fall monitoring system that protects the privacy and does not monitor a person's activities is needed. An ultrasonic-based sensor system for elderly fall monitoring in a smart room is proposed in this study. An array of ultrasonic sensors, whose ranges are designed to cover the room space, are initially installed on a wall of the room, and the sensors are rotated to transmit and receive ultrasonic signals to measure the distances to a moving object while preventing ultrasonic signal interference. Distance changes measured by ultrasonic sensors are used as time-independent patterns to recognize when an elderly person falls. To evaluate the performance of the proposed system, a sensor system prototype using long short-term memory was constructed, and experiments with 25 participants were performed. An accuracy of approximately 98% was achieved in this experiment using the proposed method, which was a slight improvement over that of the conventional method.

## 1. Introduction

The world population, which was approximately 7.7 billion people in mid-2019, is gradually increased [1]. The number of elderly people will dramatically rise to approximately 11.1%–18.6% of the total population in the next 30 years [2] due to successful birth control policies and advanced medical care services. As a result, the ratio of the working population to the elderly population is rapidly decreasing. This will lead to a worldwide labor shortage for many industries, including elderly care. At the beginning of the twenty-first century, the European commissioner launched a project called the TeleCARE consortium [3] to design and develop a virtual community infrastructure platform for elderly support. Many other countries in other regions also launched similar projects.

In the community infrastructure, the bedroom, living room, and restroom are the main rooms where elderly people spend most of their time, especially when they are at home, and it is assumed that during this time, privacy is preferred [4]. As elderly individuals are more susceptible to fatal fall [5], they need immediate assistance when a fall occurs. Therefore, automatic fall detection and alarm systems, which are used instead of caregivers to continuously monitor elderly individuals in rooms, must be developed under the conditions of privacy and trust.

The authors of this study proposed the development of an elderly fall monitoring system that can be installed in a private room. The basic conditions of this system include trust, privacy, and safety. We attempted to utilize ultrasonic sensor arrays installed on the ceiling and walls of a room to detect human falls, and experiments were performed with a static model [6–8]. A small room (30 × 30 cm^2^) with nine ultrasonic sensors was used to test the static model [6]. Ultrasonic interference between neighboring sensors and sensor calibration were found to be problems. These problems were considered, and the sensors were adjusted to mitigate interference [7]. However, coverage gaps between neighboring sensors in the array were found. The overlap of neighboring sensors was proposed to address these gaps, and experiments were performed using the model in a larger room (60 × 60 cm^2^) [8]. It was confirmed that the methods proposed in this study could be used to recognize falls using a static model. We also attempted to construct a prototype system for human fall detection. The duration of a fall is approximately 0.7 s. Accordingly, the system must be improved to be able to complete all required processes during this short period of time. Therefore, we reconsidered the system with respect to the hardware and software, improved the hardware, installed an ultrasonic sensor on a sidewall, and developed an algorithm to sense distances to humans in a point-by-point manner to detect falls using the state transition concept without identifying the specific behaviors of the person.

This study is organized as follows. The related works and smart room scenario, including the analysis of ultrasonic array sensors, are presented in Sections 2 and 3, respectively. Our proposed design method is described in Section 3. Experiments and results are reported in Section 4, and a discussion is presented in Section 5. Finally, the study is concluded in Section 6.

## 2. Related Works

Based on the research problem of elderly fall detection, many researchers have attempted to develop algorithms and systems to monitor elderly individuals and detect their falls. As shown in Table 1, research works related to the development of fall detection systems are generally divided into three approaches [37, 38]: vision-based approaches [14–20, 39–41], wearable device approaches [21–38], and ambience sensor approaches [6–8, 39–41, 42–69]. The vision-based approach is considered an excellent approach due to the beneficial 3D shape information it provides. Accurate results have also been achieved using the wearable device approach because of the dynamic personal position information obtained. Due to the sensors and their locations, sensed information using ambience sensor approaches is mainly a point-to-point approach, which is a limitation. However, the methods in this group were not originally utilized to clearly recognize an object shape. Therefore, these methods are considered to better protect resident privacy.

Previous fall detection systems using ambience devices, including infrared (IR) [39–41], IR and ultrasonic [42, 43], radar [44–51], Wi-Fi [52–57], sound [58–62], and ultrasonic [49–55] systems, have been developed, and their advantages and disadvantages are discussed as follows. IR is mainly used to confirm the absence of objects [39–41, 42, 43], but it cannot be used to measure distance, which makes 3D reconstruction difficult. Moreover, IR has been proven to be harmful to the human eyes and body [39–41, 42, 43]. As it is widely used, Wi-Fi is convenient. Radar is an excellent technique for scanning moving objects for a long time. However, both Wi-Fi and radar operate at high frequencies, which harm the human body and especially affect heart attack patients who use pacemakers [63, 64].

Other than the hearable frequency range, which causes noise harm, sound does not cause any serious harm to the human body. Furthermore, the humans cannot hear an ultrasonic sound. Therefore, sound can be safely used to measure distance using its reflected wavelength [65]. As ultrasonic sound is comparatively safe for the human body, it is recommended in this study as a good technology to develop an automatic fall detection system. In fact, ultrasonic signals, which are mainly applied in point-to-point distance measurements by directional characters, currently cannot be developed at a high resolution for object recognition due to the constraints of its beam. This observation is conversely a merit for this research problem, since, in general, elderly people prefer privacy in their living environment. The ultrasonic sensor becomes a solution to the research problem.

In the research and development of the automatic fall detection systems related to ultrasonic sensors, as shown in Table 2, Toshio Hori et al. [66] presented ultrasonic sensors, which utilized the speed of falling in a vertical direction, for elderly people and their caregivers in a nursing home. This method worked, especially in vertical falling applications, but might not be suitable for some complicated cases of diagonal falling, which is a limitation. Yirui Huang et al. [67] suggested a method to detect falls and remote activity using ultrasonic sensors. This work focused on a cost-effective and intelligent hardware design for individual ultrasonic sensors. This method also utilized the speed and level of falling in each sensor so that it was not matched with complicated fall patterns. Chang and Shih [68] proposed human fall detection based on event pattern matching with ultrasonic array sensors. This method may be used to detect many human fall patterns. However, the sensors were installed at the height of the human leg, which may not be robust enough to detect all fall patterns. Ghosh et al. [69] proposed UltraSense, which is used to identify human activity using a heterogenous ultrasonic sensor grid for smart home environments. This system identified human activity well, which is not preferred from a privacy viewpoint. Moreover, the ultrasonic sensor grid was installed on the ceiling of the room. Since height information is used, the difference between a fall and some normal activities in the vertical direction may confuse the system.

## 3. Smart Room Scenario

According to statistical data from the United Nations (UN) in 2019 [70], all societies in the world are in the midst of a “longevity revolution,” and the number of elderly people worldwide has dramatically increased year by year. In addition, children and relatives who may closely care for elderly family members do not reside with them in the same household. Approximately half of adults aged 60 and older live alone and approximately one-third live with a spouse only (without children or relatives) in North America and Europe [71]. When an elderly person on their own has a vital accident, such as a fall, it is difficult to obtain assistance as other people may not have noticed that the accident occurred. Unless someone notices and helps the person in a timely manner, an unexpected death may occur.

To solve this problem, an automatic monitoring system that protects user privacy and does not monitor activities should be installed in every house. In addition, the system must provide an immediate alert whenever a fall occurs. In our proposed scenario, an automatic monitoring system, with sensors and devices that do not directly visually recognize and record activities, is installed on the wall of a room. Therefore, an ultrasonic node was selected as the sensor in this study to continuously measure distances from the ultrasonic nodes to the person in the room in a point-to-point manner. In addition, external memory, which can store data permanently, is not utilized in this system to protect activity data. As shown in Figure 1, the fall monitoring system consists of a processor, microcontroller, and sensors that are installed in a room, which is called a smart room in this study. The system may immediately alert caregivers, relatives, and children via Wi-Fi, the cloud, and mobile phones whenever a fall occurs.

Based on the scenario of a smart room for elderly people, privacy-based and distance-based human fall detection and sensor blind zone are analyzed as follows.

### 3.1. Privacy-Based Human Fall Detection

According to the studies in [72], the human body comprises moving-independent parts or modules, and a point located on a module called a control point can represent the module position, as shown on the right side of Figure 1. If a control point representing a module is detected and the distances from the sensors to the control points are measured, the body of a person is detected and monitored. If all control points of the person are continuously detected and the distances are measured all the time, then the person's behavior is also monitored. Therefore, the patterns of control points when a fall occurs (e.g., a forward fall, a backward fall, a sideway fall, and a fall from a chair) can be observed and analyzed, as shown in Figure 2. These patterns can be trained in advance and can possibly be used to recognize falls in elderly fall monitoring systems. Although the control points of a person do not show real pictures such as a video clip captured by a closed-circuit television (CCTV), it may be possible to estimate the behaviors of the person even by the control point image. Elderly people may prefer that activities done during their private time are not monitored, as an absolute condition to develop the fall monitoring system.

Suppose that a video clip and an image of control points of humans are not allowed to be used as input data in the fall monitoring system. Instead, a point representing human body movement per frame, which contains the least amount of data in a frame and from which, it is almost impossible to determine activities, should be considered to enable fall recognition. During a fall, a point that is closest to a sensor is sensed, and this sensor may change based on the movement of the falling person. Distances from those points closest to a sensor that is continuously collecting information during a fall can be categorized into patterns based on the type of fall. Figures 3(a)–3(d) show some examples of video frames (upper row) and distances between sensors and a person (represented as a graph). The distance changes during a fall based on different fall types, e.g., forward, backward, and sideway falls and a fall from a chair, can be differentiated as patterns in the graph. These different patterns can be used to classify a fall and a nonfall as well as recognize fall types. If a classifier is trained with these distance change patterns in advance, pattern matching between these trained patterns and input data can always be used to classify the input as either a fall or a nonfall.

### 3.2. Distance-Based Human Fall Detection

To apply the abovementioned concept to the human fall problem, since the time period for a human fall is as short as approximately 0.7 s [72], the whole room space should be sensed and monitored so that the fall detection system can be processed and an alarm immediately activated during this period. In the case that a distance sensor is installed on a sidewall to measure the shortest distance from a sensor to a human at a point (*s*) in the room space, as shown in Figure 4, the change in measured distances during the fall duration (*T*_*fl*_) is mathematically expressed as the following fall pattern (*F*).

(1) $$\begin{array}{c} F=\overset{T_{fl}}{\underset{t=0}{\int }}f\left(s_{t}\right)\;dt. \end{array}$$

To cover the whole room space with ultrasonic signals without interference, multiple sensors are installed in an orderly manner in a matrix form, as shown in Figure 5. In this case, coverage ranges almost cover the sensing wall, but blind spaces or gaps exist between neighboring cells. To fill in the blind spaces, ultrasonic nodes should be shifted in an orderly manner along a straight line and simultaneously the given distance between consecutive ultrasonic nodes should be maintained to prevent interference, as shown in Figure 6(a). Additionally, the sensors can also be shifted in zigzag scanning lines to maintain balance in the horizontal and vertical directions. As an example, an ultrasonic node or more than one ultrasonic node can be scanned along a zigzag line, as illustrated by the black and red dashed arrows in Figure 6(b).

Therefore, a human fall pattern can be expressed by distance changes during a fall:

(2) $$\begin{array}{c} F=\overset{T_{fl}}{\underset{t=0}{\int }}\overset{N-1}{\underset{n=0}{\int }}\overset{M-1}{\underset{m=0}{\int }}f\left(s_{mn}\right)\;dmdndt, \end{array}$$

where *m* and *n* are the ultrasonic node positions in the horizontal and vertical directions, respectively, and *T*_*fl*_ is the human fall duration.

This fall pattern can then be converted into a digital form to realize the results using a digital computer.

(3) $$\begin{array}{c} F=\;{\left\{\overset{N-1}{\underset{n=0}{\sum }}\overset{M-1}{\underset{m=0}{\sum }}f\left(s_{mn}\right)\right\}}_{t=0}^{T_{fl}}. \end{array}$$

### 3.3. Geometric Concept for Sensor Array Installation

From the basic condition of the ultrasonic signal application, which must be generated without interference, the coverage range (*k*) on the sensing wall, as shown in Figure 7, can be obtained:

(4) $$\begin{array}{c} k=2l\cos\frac{\theta }{2}, \end{array}$$

where *l* and *θ* are the room width and sensor transmission angle, respectively.

The coverage range can be used to determine the number of ultrasonic generating nodes in the first static step (*t*_*1*_). Since it is assumed that nodes were shifted to cover all blind zones on the wall as previously described, the distance between a pair of ultrasonic sensor nodes will be calculated based on the condition of an unavoidable blind zone (*B*), as shown in Figure 8.

To apply this concept in fall detection applications, users should consider setting blind zones between consecutive ultrasonic rays at a distance smaller than the width of the human as the design condition. This guarantees the detection of human falls even in a blind zone. Thus, the range (*d*) between consecutive ultrasonic nodes can be obtained.

(5) $$\begin{array}{c} d=\frac{B\times 2cos\left(90-\theta /2\right)}{cos\left(\theta /2\right)}. \end{array}$$

In addition, the power transmitted by a string wave (*E*) can be determined as follows [73, 74]:

(6) $$\begin{array}{c} E=\frac{1}{2}\left(\mu \omega^{2}A^{2}\nu \right)=2\mu \pi^{2}f^{2}A^{2}\nu , \end{array}$$

where *μ*, *ω*, *A*, and *v* represent the mass per unit length of the string, angular frequency of the wave, wave amplitude, and wave propagation velocity, respectively.

## 4. Proposed Ultrasonic-Based Human Fall Monitoring System

Based on the abovementioned concept, a fall detection design and implementation method using ultrasonic sensors for the monitoring system is explained in this section. It is assumed that the system must be not only nonintrusive, noninvasive, and device-free but also protect the user's privacy. In the following, the system design and implementation are divided into hardware and software parts.

### 4.1. Hardware Design

The hardware system mainly consists of two units, a sensor array and a signal processing unit. The sensor array installed on a wall must be designed to cover the whole room with the smallest blind zone. In addition, the signal processing unit must provide enough ports for receiving signals from all sensors and must be designed to have enough ability to process those signals. The design of the sensor array and signal processing unit is explained as follows.

#### 4.1.1. Sensor Array

Suppose the scale of a room in which the ultrasonic sensor array for the human fall monitoring system is installed is *M* × *N* × *l*. Ultrasonic sensor nodes should be geometrically installed on a sensor wall (*M* × *N*) in the room under the condition of noninterference. The range between consecutive ultrasonic nodes in the horizontal (*φ*_*N*_) and vertical  (*φ*_*M*_) directions can be simply determined.

(7) $$\begin{array}{c} \varphi_{N}\;\geq 2l\;\tan\frac{\theta }{2},\varphi_{M}\;\geq 2l\;\tan\frac{\theta }{2}. \end{array}$$

If *B* represents the blind zone for human sensing, which has to be determined in advance, the range between consecutive sensors in the array (*d*) can be obtained based on (5).

In the first step, the number of sensors in the horizontal (*∂*_*N*_) and vertical (*∂*_M_) directions for sensing the distance in a frame, which must be limited due to the interference of ultrasonic signals from different sensors in a frame, can be simply determined.

(8) $$\begin{array}{c} \partial_{N}\geq \frac{N}{2l\;\tan\theta /2},\\ \partial_{\text{M}}\geq \frac{M}{2l\;\tan\theta /2}. \end{array}$$

Based on our proposed concept to shift the active sensors in the dense ultrasonic sensor array instead of dynamically scanning the ultrasonic sensors, the time duration for shifting mainly depends on the average human fall duration (*T*_*fl*_). If a sensing process takes a duration of time (*T*_*u*_), a shifting range (*d*), which is regarded as the dense sensor node range, can be calculated.

(9) $$\begin{array}{c} d=k/\left(\frac{T_{fl}}{T_{u}}\right). \end{array}$$

The total number of dense node sensors (*S*_*i*_) is therefore determined.

(10) $$\begin{array}{c} S_{i}=\;\frac{M\times N}{d^{2}}. \end{array}$$

#### 4.1.2. Signal Processing Unit

The signal processing unit consists of a power supply unit, an ultrasonic sensor array, a microprocessor, memory, and a classifier, as shown in Figure 8. The ultrasonic sensor array, which is supplied power by the power supply unit, always senses a moving object in the room. Analog signals representing the distance from ultrasonic sensors to a moving object are transmitted to the microprocessor. In the microprocessor, the analog signals are translated into distance data and stored in terms of a matrix in the memory. The matrix of distance data is finally fed to the classifier as a feature for fall classification.

In the power supply unit, the power needed to drive an ultrasonic sensor can be calculated based on equation (6). In equation (6), *μ*, *f*, *A*, and *ν* can be determined as the mass per unit length of the string [75], the frequency of the ultrasonic signal (defined above the sound frequency or set to 20 kHz), the amplitude of the ultrasonic signal, and the ultrasonic velocity [76], respectively.

Since this study proposes the utilization of the change patterns of distance from the ultrasonic sensor nodes to the closest point of a person who has fallen, the ultrasonic signals should be transmitted to reflect the falling person in as many round trips as possible. The number of scanning frames (*τ*) for ultrasonic signal transmission in one second can be simply estimated:

(11) $$\begin{array}{c} \tau =\frac{1}{\left(2l/v\right)+P}, \end{array}$$

where  *v*,  *P*,  and *l* are the ultrasonic signal velocity, frequency, processing time, and room depth, respectively.

In human fall detection and classification, the number of scanning frames is one of the crucial keys to fundamentally guaranteeing quality. The number of scanning frames is practically an initial condition to design the signal processing unit. Although the more scanning frames there are, the more robust the system is, and users may select an appropriate set of devices that is normally limited by processing time. For example, the processing time of a frame is limited on an approach of real time. Thus, the number of scanning frames should be calculated in real time during the period of a human falling, which is approximately 0.7 s. Suppose users fix the number of scanning frames, the maximum processing time allowed in each frame is what users may need next to select electronic devices in the hardware design step. Thus, users can expect to be able to select devices by specifications based on the allowed processing time. The processing time per frame (*P*) of devices allowed in the system design can be calculated.

(12) $$\begin{array}{c} P=\;\frac{N_{t}}{\tau }-\frac{2l}{v}, \end{array}$$

where  *v*, *τ*,  and *l* are the ultrasonic signal velocity, frequency, number of scanning frames, and room depth, respectively.

### 4.2. Software Design

The software system for retrieving ultrasonic signals representing the distance to a moving object can be designed and created, as shown in Algorithm 1. First, the initialization and declaration of variables are registered for values measured by the sensors and shown in steps 2–4. Then, an infinite loop (steps 5–14) is run to read a distance value on an ultrasonic sensor, store it in a matrix, shift the active sensor to another neighboring sensor according to the zigzag direction in Step 6 for all sensor nodes, and then classify the fall. The 2D matrix of distances in Step 6 is converted into a 1D matrix in steps 7–12, and it is fed to a classifier for fall classification in Step 13. The details of the rotation of active ultrasonic sensors and fall classification are explained in Sections 4.2.1 and 4.2.2, respectively.

#### 4.2.1. Rotation of Active Ultrasonic Sensors

To implement a software unit of the fall monitoring system, multiple ultrasonic nodes in an array are expected to simultaneously sense distances from the sensors to objects. However, interferences among ultrasonic signals may occur and lead to errors in the case where coverage areas overlap. To prevent ultrasonic signal interference, coverage areas must not overlap. The possible number of ultrasonic nodes for the simultaneous distance measurement can be determined by the minimum distance between working ultrasonic nodes, as shown in equation (7). To efficiently scan ultrasonic nodes in an array by maintaining a minimum distance, zigzag scanning is recommended to balance the horizontal and vertical directions; notably, zigzag scanning is demonstrated for a pair of ultrasonic nodes in Figure 8. Suppose that a couple of scanning lines on ultrasonic nodes in an array simultaneously start from points A and B; they synchronously move along a zigzag scanning line to the next nodes, which are labeled in the same colors. If the coordinates of ultrasonic sensor nodes are represented by row (*R*), column (*C*), and current node counting (*i*), patterns of nodes moving in a couple of zigzag scanning lines (*A* and *B*) can be logically illustrated by rows (*R*_*A*_*, R*_*B*_) and columns (*C*_*A*_*, C*_*B*_) of A and B.

**Group 1 .**

Shift from the first node (represented by a scanning line A in Figure 9)

Initially, the scanning node will be shifted to the adjacent node in the edge row as initial couple nodes. This logic can be simply expressed as follows.

Pattern *a*:
   
**IF ***I* = 0 **THEN ***R*_*A*_(*i+*1) = *R*_*A*_(*i*)*, C*_*A*_(*i+*1) = *C*_*A*_(*i*) + 1,//A : Shift straight right. *R*_*B*_(*i+*1) = *R*_*B*_(*i*) + 1*, C*_*B*_(*i+*1) = *C*_*B*_(*i*) *–* 1.//B : Shift diagonally left down

**Group 2 .**

Cases where the current sensing node is located in the 0th row (*R*_*A*_(*i*) = 0); Subgroup 2.1 Shift in the diagonal down direction (b on scanning line A in Figure 9)

When the previous sensing node (*R*_*A*_(*i–*1)*, C*_*A*_(*i–*1)) located in the 0th row is shifted right to the current sensing node (*R*_*A*_(*i*), *C*_*A*_(*i*)) located in the 0th column, the next sensing node (*R*(*i*+1), *C*(*i*+1)) will be shifted down in the diagonal direction. This logic can be expressed as follows.

Pattern *b*:
   
**IF** {*R*_*A*_*(i)* = 0} and {|*R*_*A*_*(i)*– *R*_*A*_*(i–*1)*|* = even} and {|*C*_*A*_*(i)*– *C*_*A*_*(i–*1*)|* = odd}
   
**THEN ***R*_*A*_*(i+*1) = *R*_*A*_*(i)* *+* 1*, C*_*A*_*(i+*1) = *C*_*A*_*(i) –* 1,//Shift diagonally left down
   
*R*_*B*_(*i*+1) = *R*_*B*_(*i*), *C*_*B*_(*i*+1) = *C*_*B*_(*i*) +  1.//Shift right

Subgroup 2.2. Shift right on the 0th row (f on scanning line A in Figure 9)

When the previous sensing node (*R*_*A*_(*i–*1), *C*_*A*_(*i–*1)) located outside of the 0th row approaches the current sensing node (*R*_*A*_(*i*)*, C*_*A*_(*i*)), the next sensing node (*R*_*A*_(*i+*1)*, C*_*A*_(*i+*1)) will be shifted right on the 0th row. This logic can be expressed as follows.

Pattern *c*:
   
**IF** {*R*_*A*_*(i)* = 0} and {|*R*_*A*_*(i)*– *R*_*A*_*(i–*1*)|* = even} and {|*C*_*A*_*(i)*– *C*_*A*_*(i–*1*)|* = odd}
   
**THEN ***R*_*A*_*(i+*1) = *R*_*A*_*(i), C*_*A*_*(i+*1) = *C*_*A*_*(i)* *+* 1,//Shift right
   
*R*_*B*_*(i* *+* 1) = *R*_*B*_*(i)* *+* 1*, C*_*B*_*(i+*1) = *C*_*B*_*(i) –* 1.//Shift diagonally left down

**Group 3 .**

Cases where the current sensing node is located in the 0th column (*C*_A_(*i*) = 0); Subgroup 3.1 Shift down on the 0th column (c on scanning line A in Figure 9)

When the previous sensing node (*R*(*i–*1), *C*(*i–*1)) located out of the 0th column approaches the current sensing node (*R*(*i*), *C*(*i*)) located on the 0th column, the next sensing node (*R*(*i*+1), *C*(*i*+1)) will be shifted down on the 0th column. This logic can be expressed as follows.

Pattern *d*:
   
**IF** {*C*_*A*_(*i*) = 0} and {|*R*_*A*_(*i*) *– R*_*A*_(*i–*1)| = odd} and {|*C*_*A*_(*i*) *– C*_*A*_(*i–*1)| = even}
   
**THEN ***R*_*A*_(*i+*1) = *R*_*A*_(*i+*1), *C*_*A*_(*i+*1) = *C*_*A*_(*i*),//Shift down
   
*R*_*B*_(*i+*1) = *R*_*B*_(*i*) *–* 1*, C*_*B*_(*i+*1) = *C*_*B*_(*i*) +  1.//Shift diagonally

Shift in diagonal right up direction (d on scanning line A in Figure 9)

When the previous sensing node (*R*(*i–*1), *C*(*i–*1)) located out of the 0th column is shifted down to the current sensing node (R(*i*), *C*(*i*)) located on the 0th column, the next sensing node (*R*(*i*+1), *C*(*i*+1)) will be shifted up in the diagonal direction. This logic can be expressed as follows.

Pattern *e*:
   
**IF** {*C*_*A*_(*i*) = 0} and {|*R*_*A*_(*i*) *– R*_*A*_(*i–*1)| = odd} and {|*C*_*A*_(*i*) *– C*_*A*_(*i–*1)| = even}
   
**THEN ***R*_*A*_(*i+*1) = *R*_*A*_(*i*) *–* 1*, C*_*A*_(*i*+1) = *C*_*A*_(*i*) +  1,//Shift diagonally
   
*R*_*B*_(*i*+1) = *R*_*B*_(*i*) – 1*, C*_*B*_(*i*+1) = *C*_*B*_(*i*) +  1.//Shift diagonally right

**Group 4 .**

Cases where the current sensing node is not located on the edge (*C*_*A*_(*i*)) ≠ 0 and (*R*_*A*_(*i*)) ≠ 0; Subgroup 4.1 Shift in the diagonal right direction (e on scanning line A in Figure 9)

When the previous sensing node *(R*_*A*_(*i–*1)), *C*_*A*_(*i–*1)) is shifted diagonal right up to the current sensing node (*R*_*A*_(*i*), *C*_*A*_(*i*)) located out of the 0th column and out of the 0th row, the next sensing node (*R*_*A*_(*i*+1), *C*_*A*_(*i+*1)) will be shifted up in the diagonal direction. The logic can be expressed as follows.

Pattern *f*:
   
**I**F {CA(*i*) ≠ 0} and {RA(*i*) ≠ 0} and {|RA(*i*) – RA(i–1)| = odd}and{|CA(*i*) – CA(i–1)| = odd}
    THEN RA(*i*+1) = RA(*i*) – 1, CA(*i*+1) = CA(*i*) +  1,//Shift diagonally up. RB(*i*+1) = RB(*i*) +  1, CB(*i*+1) = CB(*i*).//Shift down

Subgroup 4.2. Shift in the diagonal left direction

When the previous sensing node (RA(i–1), CA(i–1)) is shifted diagonal right up to the current sensing node (RA(*i*), CA(*i*)) located out of the 0th column and out of the 0th row, the next sensing node (RA(*i*+1), CA(*i*+1)) will be shifted down in the diagonal direction. This logic can be expressed as follows.

Pattern g:
   
**IF** {*C*_*A*_(*i*) ≠ 0} and {*R*_*A*_(*i*) ≠ 0} and {|*R*_*A*_(*i*) – *R*_*A*_(*i–*1)| = odd} and {|*C*_*A*_(*i*) *– C*_*A*_(*i–*1)*|* = odd}
   
**THEN ***R*_*A*_(*i*+1) = *R*_*A*_(*i*) +  1*, C*_*A*_(*i+*1) = *C*_*A*_(*i*) – 1,//Shift diagonally left down. RB(*i*+1) = RB(*i*) – 1, CB(*i*+1) = CB(*i*) +  1.//Shift diagonally right up

These logics cover the possible movement of a couple of current sensing nodes (*R*_*A*_(*i*), *C*_*A*_(*i*)) and (*R*_*B*_(*i*), *C*_*B*_(*i*)) to the next sensing nodes (*R*_*A*_(*i*+1), *C*_*A*_(*i*+1)) and (*R*_*B*_(*i+1*)*, C*_*B*_(*i* *+* 1)) in a couple of zigzag scanning lines. As an example, an algorithm for shifting a couple of sensing nodes to the next sensing nodes in a couple of zigzag scanning lines is described in Algorithm 2.

#### 4.2.2. Fall Classification

Due to the time limitation and time invariance of a human fall, long short-term memory (LSTM), which is regarded as an excellent classifier for time invariance, is utilized in this study. Distance information from sensors to a human is assumed to be input data for the classifier. As shown in Figure 10, the node number in the input layer is determined based on the number of sensors that sense a moving object during a human fall, which is assumed to take approximately 0.7 s, and the output nodes for the fall detection system should be set as many to one, with a number of preference choices, such as a backward fall, forward fall, or walking. The hidden layer of the LSTM is used to set the input size per series to 2/3 of its original value [77].

Pretests must be performed on some samples using possible parameters in the training state to determine the experimental parameter settings. As shown in Table 3, the activation function (e.g., softmax, ReLU, sigmoid, and tanh) should be pretested on some samples in advance and selected appropriately for the networks. In the input layer, the batch size, input size per series, input feature, and learning rate are trained with a number of 2^n^ within the capability of the graphics processing unit (GPU) memory, total number of input data of all features, input data dimension, and appropriate rate for gradient descent that considers an appropriate time, respectively, without overshooting [78].

## 5. Experiments and Results

To evaluate the performance of the proposed method, a room with ultrasonic sensors installed was constructed, and a data processing system was implemented based on the experimental specifications, as shown in Table 4. For the experiments, a representative group of participants were selected based on sex and age. These participants were trained to walk, sit, and fall in the room before experiments were performed. The LSTM classifier was set up based on the specifications shown in Tables 1 and 2. Photographs of an empty room, a room with a participant, and our design interface with a memory card are shown in Figures 11(a)–11(c), respectively. The experiments were performed by 25 participants using some behavior criteria, including falling, walking, and sitting in the constructed room, as shown in Table 5. The experimental results obtained in distance data of one and two points per frame reveal the human fall recognition rate based on the number of training and testing samples, as shown in Tables 6 and 7, respectively. The results are divided into the following groups: 20–40 years of age and 41 years of age and older. Training and testing data from the experiment were processed with ratios of 90 : 10, 80 : 20, 70 : 30, 60 : 40, and 50 : 50 to access the accuracy of the training and testing criteria. An accuracy of approximately 99.14% was achieved using the ratio of 90 : 10 after the training and testing experiments. Compared with conventional methods, the proposed method exhibited an improvement in accuracy by approximately 1.14%, as shown in Table 8. Examples of distances captured by two node sensors in the cases of a forward fall, backward fall, fall from a chair, and walking during 1,000 ms are shown in Figure 12. These graphs show patterns of distance changes for each case. While ultrasonic signal transmitters are located on a wall scan in the zigzag direction to transmit ultrasonic signals by two nodes each time, distances are always measured by 16 sensors (0,0–3,3) located on the opposite sidewall. All measured distances during 1,000 ms are shown in the graphs. In these measured distance data, differences among a forward fall, backward fall, sideway fall, fall from a chair, and walking were observed. These data were input into the LSTM for training and classification.

In the experiments, the measured distances in continuing frames that showed behaviors, such as falling, walking, and sitting done by the 25 participants (as shown in Table 4), were used to train and test with various ratios. Errors occurred based on the use of one node or two nodes, as shown in Table 9, respectively (Table 10). These errors are analyzed in the discussion.

## 6. Discussion

To build a smart room that can be used to detect the falls of elderly people without an intrusion of privacy, this study proposes installing an array of ultrasonic sensors on a wall, activating the sensors to sense distance information, and classifying the falls of elderly people based on distance change patterns. The performance of the proposed method was evaluated, and the accuracy was more than 90% in the cases of training more than 50% of the 2 node-based sample data, as shown in Table 7. Based on the results of the 1 node-based data shown in Table 6, the accuracy using this method was worse than that of the 2 node-based data because sensing based on one node was insufficient to cover the whole room. If the room was much smaller so that the range of the ultrasonic signal covered the room, one node would be adequate. Users must consider the coverage range of the ultrasonic signals with respect to the room scale as one of the design conditions. The results shown in Tables 5 and 6 confirm the effective range of sensor coverage and were used to evaluate the performance of the proposed method. Acceptable accuracy was achieved. The accuracy increased according to the increasing ratio of training samples, and an approximately 98% accuracy was achieved using the 90 : 10 training and testing ratio. Although elderly individuals (individuals over 40 years of age in this experiment) comprehensively caused both positive and negative faults, they contributed a large number of true positives to the results compared with the other group. Therefore, the proposed method was considered to be applicable to elderly individuals. The proposed method was compared with conventional methods, and it was obvious that higher precision and recall were obtained using the proposed method, as shown in Table 8. These high accuracy results were analytically caused by the distance change patterns of forward, backward, and sideway falls, falls from a chair, and especially walking, as shown by the examples in Figure 12. As observed change patterns among consecutive frames in the time domain, classifiers for video were confirmed to be appropriate tools for this kind of fall detection and classification problem. Analytically, errors decreased when the number of training samples was increased compared with testing samples, and accuracy was considered reliable in the 90 : 10 training and testing ratio, as shown in Tables 9 and 10. Therefore, the proposed method was proven to be effective for fall classification.

In addition, the fault-positive (FP) and fault-negative (FN) errors shown in the middle column of Tables 6 and 7 were analyzed, and causes of these errors were found, as shown in Table 11. The FP column in Table 10 indicates the number of positive errors in many error patterns, such as misclassifying sitting as falling and misclassifying the type of fall. These errors may cause a caregiver to be alerted to provide help to an elderly person who has fallen. Although these errors were considered a waste of time and energy for the caregivers, they were counted as positive errors and were considered a safety measure. However, the FN column in Table 11 indicates some cases of falling from a chair that were misclassified as sitting on a chair. After analyzing the photographs and signals of this case, as shown by the examples in Figure 13, respectively, and Figure 14, the video shots and signal patterns that represented falling and sitting looked similar and were hard to differentiate, even when judged by human eyes. This result was considered a limitation of the proposed method. Additional features, such as distance changes measured from the roof, should be considered as future work to solve this limitation. An additional limitation was that an ultrasonic signal was transmitted from a node as a triangular shape, as observed from the top view. Therefore, small areas between neighboring nodes were regarded as blind areas in which falls were impossible to detect. System designers must carefully design the number of ultrasonic nodes in the array based on the blind zone to be smaller than the minimum human width, as recommended above. This may guarantee protection against not detecting a human fall.

## 7. Conclusions

To prevent serious risks to elderly individuals after falling in a room, it is necessary to simultaneously monitor elderly behaviors without intruding on their privacy, detect falls, and immediately inform caregivers, when a fall occurs so they can provide urgent assistance. A design method for an ultrasonic sensor-based system is proposed in this study for elderly fall monitoring in a smart room. In this design, ultrasonic sensors are installed as a sensor array on a wall under the condition that the ultrasonic signal covers the area of the whole room with a limited blind zone. The blind zone is determined in advance to be smaller than the width of the human, and the determined blind zone and average human fall duration are used to calculate the distance between neighboring ultrasonic nodes and the total number of ultrasonic nodes on a wall. Then, activated ultrasonic nodes are transmitted in a one-by-one manner without interference in a zigzag scanning line, and the ultrasonic signals, which are time-independent, are classified as a fall or a nonfall by a time-independent-based classifier, such as LSTM. The performance of the proposed method is confirmed to be effective.

## Figures and Tables

**Figure 1:** A human body and its control points sensed by a sensor array.

**Figure 2:** Control points during falls. (a) A forward fall. (b) A backward fall. (c) A sideway fall. (d) A fall from a chair.

**Figure 3:** Distance patterns during falls. (a) Pattern of a forward fall. (b) Pattern of a backward fall. (c) Pattern of a sideway fall. (d) Pattern of a fall from a chair.

**Figure 4:** Pattern of distance changes.

**Figure 5:** Distance sensing matrix.

**Figure 6:** Scanning lines: (a) straight lines and (b) zigzag lines.

**Figure 7:** Coverage and shifting ranges.

**Figure 8:** Signal processing unit.

**Figure 9:** Zigzag scanning patterns for a pair of ultrasonic nodes.

**Figure 10:** Long short-term memory for classification.

**Figure 11:** Photographs of the experiments.

**Figure 12:** Distances in fall cases: (a) forward fall, (b) backward fall, (c) sideway fall, (d) fall from a chair, and (e) walking.

**Figure 13:** Photographs representing the system misclassification of falling as sitting: (a) sitting on a chair and (b) falling from a chair.

**Figure 14:** Similar distance change patterns of sitting and falling.

**Algorithm 1:** Comprehensive system of the proposed fall detection and classification.

**Algorithm 2:** Zigzag scanning.

**Table 1:** Research works related to image-based and wearable fall detection systems.

Algorithm name	Sensor and equipment	Feature extraction technique	Classification algorithm	Accuracy/error
1. Image-based fall detection systems				
Hernandez [11]	2D camera and OpenCV	Rectangle enclosing	Threshold-based	Accuracy 85.37%
Lin [12]	GMM and MHI	Acceleration and angular acceleration	Accurately model an ellipse	—
Basavaraj [13]	MHI and ellipse approximation	Both ellipse approximation and MHI	Accurately model an ellipse	Accuracy 86.66%
ShanShan [14]	Semi-contour distances	Points on the vertical line	SVM	—
Chen [15]	Depth camera	Histogram of oriented gradient (HOG)	SVM and ANN	Sensitivity 77.98%, specificity 87.58%, accuracy 82.84
Cai [16]	Optical flow combining with wide residual network	Optical flow and residual network	Softmax classifier	Accuracy 92.6%
Marcos [17]	Transfer learning, optical flow algorithm	Displacement vector optical flow algorithm	Fully connected neural network	Sensitivity 95%, specificity 96%
Lu [18]	3D CNN was used	Temporal motion feature, 3D CNN	SVM	Accuracy 99.3%
Miguel [19]	Low-cost device, Raspberry Pi	Background subtraction Kalman filter	KNN	Sensitivity 96% specificity 97%
Lotfi [20]	Major and minor semi-axis of ellipse fitting silhouette	Spatiotemporal	Multilayer perceptron neural network	Accuracy 99.2%, sensitivity 99.5%, specificity 97.3%
2. Wearable fall detection systems				
Freitas [21]	BLE module and a microprocessor	Acceleration	Fall signal to Web app	—
Pierleoni [22]	Magnetic, angular rate, and gravity (MARG) sensor	Yaw, pitch, and roll, Madgwick orientation filter	Threshold and SVM	Accuracy 90.37%, sensitivity 80.74%
Otanasap [23]	Using tri-dimensional accelerometer	Acceleration, ADL value	Dynamic threshold model	Accuracy 97.40%, sensitivity 99.48%
Kurniawan [24]	Using tri-dimensional accelerometer	Yaw, pitch, and roll, alpha	SVM	Accuracy fall forward 95%, accuracy fall backward 75%
Chu [25]	Wearable device that combined BLE	Acceleration	Exponential smoothing gray model (ESGM)	—
Shahiduzzaman [26]	Smart helmet	Biomedical sensing data	SVM	Accuracy 96.67%
Nari [27]	Accelerometer and gyroscope	ACC and gyro	Threshold-based	Sensitivity 90% and specificity 86.7%
Nho [28]	Heart rate sensor and accelerometer	Cluster analysis-based user-adaptive fall detection	Fourfold cross-validation, 13-dimensional	Accuracy 97.51%, sensitivity 99.17%
Chen [29]	Crowdsourcing-based adaptive datasets	Acceleration, inclination angle	Threshold-based	Accuracy 97%
Tang [30]	Radar sensors on shoe	Distance-to-obstacle	Threshold-based	—
Djelouat [31]	Compressed sensing	Acceleration	Extended nearest neighbor	Accuracy 91.73%
Jahanjoo [32]	Neural network classification algorithm	43 features, FFT, principal component analysis	Multilevel fuzzy min-max neural network	Sensitivity 97.29%, specificity 98.7%
Mao [33]	Magnetometer accelerometer gyroscope	Acceleration, Euler angle (orientation)	Threshold-based	Accuracy 100% sensitivity 100%
Ang [34]	Multiple power-saving algorithms	Acceleration	Decision tree classifier	Sensitivity 91%
Purushothaman [35]	A neural network classification algorithm	Linear and angular acceleration	Neural network	—
Khojasteh [36]	Threshold optimization	Eight features from acceleration	SVM, RBS, and DT	Accuracy 95.15%
De Quadros [37]	Madgwick's decomposition	Statistical features from acceleration	SVM-KNN with Madgwick's decomposition	Sensitivity 93%, specificity 98%
Saleh [38]	Two-segment feature extraction	Statistical 12 feature vectors from acceleration	Artificial neural network and SVM	Accuracy 99.9%, sensitivity 99.1%, specificity 99.9%

**Table 2:** Research works in ambience sensor-based systems.

Algorithm name	Sensor and equipment	Feature extraction technique	Classification algorithm	Accuracy/error
Ambience sensor-based fall detection systems				
1.1 IR sensor				
Tzeng [39]	Floor pressure and infrared image	Average image pixel value (mean)	Image thresholding	Accuracy 98.3%
Guan [40]	Infrared signal-based	Multi-sensor time	K-nearest neighbor, GM-HMM, SVM	Sensitivity 98%, specificity 93%
Ogawa [41]	IR array sensor	Temperature distribution × 20	Machine learning	Accuracy 97.75%
Asbjørn [42]	IR array sensor	80 × 60 thermal array	Multilayer perceptron model	Accuracy 96.73%
Chen [43]	Infrared arrays and ultrasonic	8 × 8-pixel thermal, RMS values	SVM	Accuracy 90.3%
1.2 Radar sensor				
*A*_min_ [44]	Real fall data used	MFCC, SWT	SVM and WT-based algorithm	—
Liu [45]	Doppler radar motion	MFCC	SVM and KNN	—
Tomii [45]	Multiple Doppler sensors	Compensates the drawbacks of mono-Doppler sensor	SVM and KNN	Accuracy 95.5%
Wu [47]	Radar signal	Pursuit decomposition, time-frequency	PCA, HMM, SVM	—
Wang [48]	Pulse Doppler radar for passive	Angle *θ* and *ϕ* affect	Walking sequence selection/speed estimation	—
Gadde [49]	Radar signal	Time scale	Wavelet transform	—
Wu [50]	Radar technology	Extreme frequency magnitude	Bayesian, SVM	—
Su [51]	Doppler radar	MFCC features	Wavelet transform	—
1.3 Wi-Fi device				
Wang [52]	Wi-Fi device	Channel state information (CSI)	SVM	Sensitivity 92%, specificity 92%
Khan [53]	Passive Wi-Fi sensing, Vi Wi	Two-dimensional phase extraction system	Tremor classification	Accuracy 98%
Gu [54]	Wi-Fi device	Channel state information (CSI)	Activity recognition	Accuracy 94.58%
Ramezani [55]	Wi-Fi, accelerometer, and floor vibration	CSI, STD, MAD, IR, SRS	SVM	—
Cheng [56]	Wi-Fi signals	Channel state information (CSI)	CNN, LSTM, GRU	—
Hu [57]	Wi-Fi	Channel state information (CSI)	SLN-DTW	Accuracy 96%
1.4 Acoustic sensor				
Zigel [58]	Acoustic signal	Pattern recognition, event segmentation	Event classification	—
Li [59]	Circular array of 8 microphones	MFCC	Nearest neighbor	AROC 0.98
Li [60]	Beamforming to increase signal strength	MFCC	Nearest neighbor	Sensitivity 100%, specificity 97%
Li [61]	8-Microphone circular array	iVAT clustering and GA-based	Nearest neighbor	—
Cheffena [62]	Smartphone	The spectrogram, MFCCs, LPC, and MP	ANN	Accuracy 98%
1.5 Ultrasonic sensor				
Yoshio [66]	Ultrasonic sensor network and floor mat sensor	Tracking a head of moving human	Pattern trajectories	—
Huang [67]	Ultrasonic sensor array, FPGA	Distance, time duration	Pattern matching	—
Chang et al. [68]	Arduino ultrasonic array	Time energy	SVM	Accuracy 98%
Nadee et al. [6]	Ultrasonic array: ceiling, sidewall	Distance, time duration	Threshold-based	Accuracy 92%
Nadee et al. [7]	Ultrasonic array: two temperature sensor error correction	Distance, time duration	Threshold-based algorithm	Accuracy 93%
Nadee et al. [8]	Ultrasonic array: octagonal array	Distance, time duration	Threshold-based algorithm	Accuracy 94%
Ghosh et al. [69]	HC-SR04, LV-Max Sonar-EZ0 sensor	Distance, time duration	Decision tree	Accuracy 90%
This work	Ultrasonic array: MaxSonar MB1010	Distance, time duration	LSTM	Accuracy 98%

**Table 3:** Classification specification.

Layer	Parameter	Value
Input	Batch size	12
	Input size per series	16
	Input feature	1 dimension
	Learning rate	0.001

Hidden layer	LSTM hidden layer	
	Hidden node	100
	Activation	

Output layer	LSTM model	
	Output class	12

**Table 4:** Experimental specifications.

Devices/software/participants	Specifications
Computer system	Aspire VX15
	CPU : Intel Core i7-7700HQ
	GPU : NVIDIA GeForce GTX 1050
	Memory size: 12 GB DDR4
	Hard disk drive: SSD 512 GB
Basic programming	MATLAB_R2019b
Participants	25 people
Age and height ranges of participants	21–30 years; male: 8; female: 2; 158–175 cm
	31–40 years; male: 4; female: 0; 165–178 cm
	41–50 years; male: 3; female: 1; 158–175 cm
	51–60 years; male: 2; female: 0; 158–175 cm
	>60 years; male: 3; female: 2; 158–175 cm
Experiment 1 (walk)	Participants: 25 people: 8 groups
Experiment 2 (fall)	Participants: 25 people: 4 groups
Room size	Size: 200 × 200 cm^2^
Sensors	16 nodes
Distance between sensors	50 cm
Blind spot distance	15.2 cm

**Table 5:** Samples for training and testing.

No.	Posture	Category	No. of samples
1	Forward fall	1	100
2	Backward fall	2	100
3	Left and right sideway falls	3	100
4	Fall from a chair	4	100
5	Walk to chair	5	25
6	Walk to sensor	6	25
7	Walk away from sensor	7	25
8	Walk in a circle	8	25
9	Walk left to right	9	25
10	Walk right to left	a	25
11	Walk diagonal left to right	b	25
12	Walk diagonal right to left	c	25
Total of samples			600

**Table 6:** Experimental results based on one node.

1 node												
Train/test	Recognition (%)	Error (%)	SD	TP			FP			FN		
				Age		Total	Age		Total	Age		Total
				20–40	>40		20–40	>40		20–40	>40	
90/10	95.74	4.26	0.52	23	34	57	1	2	3	0	0	0
80/20	89.58	10.42	0.56	43	64	107	4	6	10	1	2	3
70/30	86.43	13.57	0.63	62	94	156	7	11	18	3	4	7
60/40	79.72	20.28	0.60	77	114	191	14	24	38	5	6	11
50/50	70.33	29.67	0.65	84	127	211	24	38	62	12	15	27

**Table 7:** Experimental results based on two nodes.

2 nodes												
Train/test	Recognition (%)	Error (%)	SD	TP			FP			FN		
				Age		Total	Age		Total	Age		Total
				20–40	>40		20–40	>40		20–40	>40	
90/10	98.15	1.85	0.50	24	35	59	0	1	1	0	0	0
80/20	96.47	3.53	0.53	46	70	116	2	2	4	0	0	0
70/30	93.43	6.57	0.57	67	101	168	5	7	12	0	0	0
60/40	90.58	9.42	0.57	88	130	218	7	13	20	1	1	2
50/50	86.56	13.44	0.63	104	156	260	14	21	35	2	3	5

**Table 8:** Performance comparison with conventional methods.

Method	Recognition ratio (%)	Precision (%)	Recall (%)	SD
Huang et al. 2012 [67]	92	—	—	—
Chang et al. 2017 [68]	98	—	—	—
Ghosh et al. 2019 [69]	90	74	100	—
Proposed method	98.15	98.30	100	0.500

**Table 9:** Error analysis based on one node.

Ratio of training/testing	90:10		80:20		70:30		60:40		50:50	
Type	Correct	Error	Correct	Error	Correct	Error	Correct	Error	Correct	Error
Forward fall	10		19	1	24	6	29	11	35	15
Backward fall	10		18	2	25	5	33	7	38	12
Left and right sideway fall	10		17	3	26	4	35	5	33	17
Fall from a chair	8	2	17	3	24	6	32	8	34	16
Walk left to right	3		5		7	1	7	3	9	4
Walk right to left	2		4	1	7		7	3	9	3
Walk in a circle	3		4	1	7	1	8	2	10	3
Walk diagonal left to right	2		5		7	1	8	2	8	4
Walk diagonal right to left	3		3	2	7	1	8	2	7	6
Walk to sensor	2		5		7		7	3	9	3
Walk away from sensor	3		5		8		9	1	10	3
Walk to chair	2		5		7		8	2	9	3

Sum	58	2	107	13	156	25	191	49	211	89

**Table 10:** Error analysis based on two nodes.

Ratio of training/testing	90:10		80:20		70:30		60:40		50:50	
Type	Correct	Error	Correct	Error	Correct	Error	Correct	Error	Correct	Error
Forward fall	10		20		29	1	38	2	47	3
Backward fall	10		20		28	2	37	3	46	4
Left and right sideway fall	10		19	1	29	1	38	2	46	4
Fall from a chair	9	1	18	2	28	2	37	3	45	5
Walk left to right	3		5		7	1	8	2	10	3
Walk right to left	2		5		6	1	8	2	9	3
Walk in a circle	3		5		8		9	1	11	2
Walk diagonal left to right	2		5		6	1	8	2	9	3
Walk diagonal right to left	3		5		7	1	9	1	10	3
Walk to sensor	2		5		7		10		10	2
Walk away from sensor	3		5		7	1	8	2	9	4
Walk to chair	2		4	1	6	1	8	2	8	4

Sum	59	1	116	4	168	12	218	22	260	40

**Table 11:** Error analysis based on two nodes.

Train/test			FP		FN			
1	90/10	Correct	Beside to fall		Sum	Correct	—	—
		Error	Side fall left and right			Error	—	—
			1		1			
2	80/20	Correct	Beside to fall		Sum	Correct	—	—
		Error	Side fall left and right			Error	—	—
			2		2			
		Correct	Side fall left and right					
		Error	Beside to fall					
			1		1			
		Correct	Walk to sit					
		Error	Walk to sensor					
			1		1			
3	70/30	Correct	Side fall		Sum	Correct	—	—
		Error	Forward fall	Blackward fall		Error	—	—
			1	1	2			
		Correct	Blackward fall					
		Error	Forward fall	Side fall left and right				
			1	1	2			
		Correct	Forward fall					
		Error	Backward fall					
			1		1			
		Correct	Side fall left and right					
		Error	Beside to fall					
			1		1			
		Correct	Walk left to right					
		Error	Walk right to left					
			1		1			
		Correct	Walk right to left					
		Error	Walk left to right					
			1		1			
		Correct	Walk diagonal left to right					
		Error	Walk diagonal right to left					
			1		1			
		Correct	Walk diagonal right to left					
		Error	Walk diagonal left to right					
			1		1			
		Correct	Walkout sensor					
		Error	Walk to sensor					
			1		1			
		Correct	Walk to sit					
		Error	Walk diagonal left to right					
			1		1			
4	60/40	Correct	Side fall left and right		Sum	Correct	Walk to sit	Sum
		Error	Forward fall	Blackward fall		Error	Beside to fall	
			1	1	2		2	2
		Correct	Blackward fall					
		Error	Forward fall	Side fall left and right				
			2	1	3			
		Correct	Forward fall					
		Error	Backward fall	Side fall left and right				
			1	1	2			
		Correct	Beside to fall					
		Error	Forward fall	Side fall left and right				
			1	2	3			
		Correct	Walk left to right					
		Error	Walk right to left					
			2		2			
		Correct	Walk right to left					
		Error	Walk left to right					
			2		2			
		Correct	Walk diagonal left to right					
		Error	Walk diagonal right to left					
			1		1			
		Correct	Walk diagonal right to left					
		Error	Walk diagonal left to right					
			1		1			
		Correct	Walkout sensor					
		Error	Walk to sensor					
			2		2			
		Correct	Walk to sit					
		Error	Walk diagonal left to right					
			2		2			
5	50/50	Correct	Side fall left and right		Sum	Correct	Walk to sit	Sum
		Error	Forward fall	Beside to fall		Error	Beside to fall	
			2	2	4		3	3
		Correct	Blackward fall			Correct	Beside to fall	
		Error	Forward fall	Side fall left and right		Error	Walk to sit	
			2	2	4		2	2
		Correct	Forward fall					
		Error	Backward fall	Side fall left and right				
			1	1	2			
		Correct	Beside to fall					
		Error	Forward fall	Side fall left and right				
			1	2	3			
		Correct	Walk left to right					
		Error	Walk right to left	Walk out sensor				
			2	1	3			
		Correct	Walk right to left					
		Error	Walk left to right					
			3		3			
		Correct	Walk circle					
		Error	Forward fall	Backward fall				
			1	1	2			
		Correct	Walk diagonal left to right					
		Error	Walk diagonal right to left					
			3		3			
		Correct	Walk diagonal right to left					
		Error	Walk diagonal left to right					
			3		3			
		Correct	Walkout sensor					
		Error	Walk to sensor					
			2		2			
		Correct	Walk to sensor					
		Error	Walkout sensor	Walk right to left				
			3	1	4			
		Correct	Walk to sit					
		Error	Walk diagonal left to right					
			2		2			

## Data Availability

Data are available at https://livermutlac-my.sharepoint.com/:f:/g/personal/eleccmk_rmutl_ac_th/EsYB9mvw2ZpFiXJ9zervDcIBSBdMa3enOdK17fhf0M2-DA?e=Znch33.
